The article "Correlation and Diagnostic Value of Serum Cys-C, RBP4, and NGAL with the Condition of Patients with Traumatic Acute Kidney Injury" was retracted in 2023. Reasons: signs of a paper mill; compromised peer review; unreliable results or conclusions.

# Correlation and Diagnostic Value of Serum Cys-C, RBP4, and NGAL with the Condition of Patients with Traumatic Acute Kidney Injury

**DOI:** 10.1155/2021/4990941

**Published:** 2021-09-03

**Authors:** Zufeng Ye, Hui Liu, Bixia Zhao, Hao Fu, Ying Li, Li Chen

**Affiliations:** ^1^The Affiliated Nanhua Hospital, Department of Clinical Laboratory, Hengyang Medical School, University of South China, Hengyang, Hunan 421001, China; ^2^The Affiliated Nanhua Hospital, Department of Emergency, Hengyang Medical School, University of South China, Hengyang, Hunan 421001, China; ^3^The Affiliated Nanhua Hospital, Department of Urology, Hengyang Medical School, University of South China, Hengyang, Hunan 421001, China; ^4^The Affiliated Nanhua Hospital, Department of Anesthesiology, Hengyang Medical School, University of South China, Hengyang, Hunan 421001, China; ^5^The Affiliated Nanhua Hospital, Department of Nursing, Hengyang Medical School, University of South China, Hengyang, Hunan 421001, China

## Abstract

There is a lack of targeted biomarkers that can diagnose Acute Kidney Injury (AKI) early and accurately, which leads to deterioration of renal function and even death in patients who do not receive timely and effective treatment. In recent years, an increasing number of studies have shown that AKI-related markers such as cystatin C (Cys-C) and retinol-binding protein (RBP) can be used for early diagnosis of AKI to a certain extent. A total of 262 subjects were included in this study, of which 132 patients with traumatic AKI were enrolled in one group and named as the AKI group; 130 healthy subjects were enrolled in another group and named as the healthy group. AKI patients with different conditions were classified into AKI phase I, II, and III according to the KDIGO AKI diagnostic criteria, with 45, 59, and 28 in each group. In this study, we examined and compared serum Cys-C, RBP4, and neutrophil gelatinase-associated lipid transport protein (NGAL) levels between the AKI and healthy groups and between patients with AKI of different conditions, and the correlation and diagnostic value of three serum markers with the condition of traumatic AKI patients were also analyzed. The results showed that serum Cys-C, RBP4, and NGAL were significantly higher in the AKI group compared with the healthy group (*P* < 0.05), and the mean concentrations of the three serum markers increased as the severity of the disease increased, while correlation analysis showed that all three serum markers were positively correlated with serum Scr levels (*P* < 0.001). Further ROC curve analysis was performed, and the diagnostic values of serum Cys C, RBP4, and NGAL alone and in combination for traumatic AKI were 0.769, 0.741, 0.771, and 0.905, respectively. In short, serum Cys C, RBP4, NGAL have important value for the assessment and diagnosis of traumatic AKI patients.

## 1. Introduction

Acute kidney injury (AKI) is a common complication in patients with severe trauma, where patients suffer from tissue damage, shock, or infection that can lead to immune dysfunction and promote the release of large amounts of inflammatory factors, which in turn leads to systemic inflammatory response syndrome and multiorgan dysfunction syndrome, complicated by AKI [1]. Early detection, early diagnosis, and early treatment are the basic treatment principles for traumatic AKI. Timely and accurate diagnosis of traumatic AKI and taking appropriate measures to mitigate the progression of AKI can achieve improved patient prognosis and reduced morbidity and mortality [2, 3]. Currently, the diagnosis of traumatic AKI mainly relies on medical history, serum creatinine (Scr), and changes in its urine volume, but the diagnosis takes relatively long and the abovementioned indicators are easily interfered by other factors [4]. Therefore, we need to look for plus sensitive serum markers to determine whether AKI is present in patients with traumatic diseases.

Cystatin C (Cys-C) is a cysteine protease inhibitor that is distributed in various body fluids such as blood and cerebrospinal fluid, and its production is not affected by other physical characteristics or external conditions [5]. One study [6] noted that a significant increase in Cys-C levels could be observed in the serum of patients with AKI and correlated with the severity of kidney damage. Retinol-binding protein 4 (RBP4) is a carrier protein that exists in blood mainly as a retinol-RBP4 complex (holo-RBP). With the decline of glomerular filtration function and renal blood flow, RBP4 will accumulate in various forms and increase the blood RBP4 concentration [7, 8]. Neutrophil gelatin-related lipid transporter protein (NGAL) belongs to the superfamily of lipid transport proteins, which are not very active under normal conditions and are present in very low concentrations in the blood. However, after the onset of AKI, an increase in NGAL concentrations can be detected in the blood and urine of patients [9, 10].

The search for more sensitive serum markers associated with AKI to improve its diagnostic accuracy has been the focus of many studies. There are numerous studies on novel markers, and this article will briefly review the relevance and diagnostic value of Cys-C, RBP4, and NGAL in patients with traumatic AKI.

## 2. Information and Methods

### 2.1. Baseline Information

132 patients with traumatic AKI admitted to our hospital between January 2017 and December 2019 were selected as the AKI group. Causes of injury: 46 cases of traffic accidents, 34 cases of falling from heights, 25 cases of mechanical strangulation, 16 cases of heavy object injury, 8 cases of knife stabbing, 2 cases of engineering accident injury, and 1 case of gunpowder gunshot injury. The patients with traumatic AKI were classified into AKI phase I (45 cases), AKI phase II (59 cases), and AKI phase III (28 cases) according to the KDIGO AKI diagnostic criteria. In addition, we also selected 130 subjects who underwent health checkups at our hospital during the same period as the health group. The comparison of baseline information between the AKI group and the healthy group is shown in Figure 1 and Table 1.

### 2.2. The Inclusion Criteria

(1) Patients with rapidly declining renal function within 48 h, with an absolute increase in Scr ≥26.5 *μ*mol/l or ≥50% increase from basal values or urine output <0.5 ml/(kg·h) for more than 6 hours. (2) Patients who had a clear history of trauma. (3) The patient or family has signed an informed consent form.

### 2.3. The Exclusion Criteria

(1) Patients with severe failure of other organs such as the heart, liver, and spleen. (2) Patients who have used hormone therapy within the last 1 month. (3) AKI due to nontraumatic diseases. (4) Patients with kidney tumors. (5) Patients with primary kidney disease or urinary tract infection, those with diabetic nephropathy, those with acute and chronic renal failure due to other causes such as nonsevere trauma, and those with a history of renal transplantation. (6) Patients with incomplete clinical information.

### 2.4. The Specific AKI Phasing Criteria [11]

An elevation in Scr of 1.5 to 1.9 times the baseline value or an elevated value ≥26.5 *μ*mol/l and/or a urine volume <0.5 ml/(kg·h) for 6 to 12 hours was considered AKI phase I. Scr elevation of 2 to 2.9 times the baseline value and/or urine volume <0.5 ml/(kg·h) for ≥12 hours was considered AKI phase II. Scr increased more than 3 times the baseline value or increased ≥353.6 *μ*mol/l or required renal replacement therapy and (or) urine output <0.3 ml/(kg·h), lasting ≥24 h, or the absence of urine for ≥12 hours was considered AKI phase III.

### 2.5. Research Method

#### 2.5.1. Major Reagents and Instruments

The Serum Cys-C ELISA Kit, Serum RBP4 ELISA Kit, and Serum NGAL ELISA Kit (Shanghai Yuanmu Biotechnology Co., Ltd.); BK-400 Automatic Biochemical Analyzer (Shandong Boke Biological Industry Co., Ltd.); Centrifuge (Jiangsu Zhengji Instrument Co., Ltd.); and Enzyme Labeler (Bio-Rad Corporation, USA) were used.

#### 2.5.2. Testing Method

In the AKI group, 5 mL of peripheral venous blood was collected with a sodium citrate vacuum anticoagulation tube immediately after admission to the hospital at the time of diagnosis of traumatic AKI. Patients in the healthy group were collected at the time of physical examination, and the blood specimens were centrifuged at 2000 r/min for 20 min at room temperature and separated from the plasma specimens, which were numbered and stored in liquid nitrogen filling for testing. The enzyme-linked immunosorbent assay (ELISA) was used to detect the levels of serum Cys-C, RBP4, and NGAL. The experimental steps included dilution and addition of standards, addition of samples, warming, preparation, washing, enzyme addition, warming, washing, color development, termination, and determination. The specific operations were carried out strictly according to the kit instructions. The determination was carried out within 15 minutes after the addition of the stop reagent. The absorbance (OD) of each well was measured sequentially at 450 mm wavelength using an enzyme marker, and the concentration corresponding to the sample to be measured was calculated according to the standard curve.

### 2.6. Statistical Methods

SPSS 20.0 software was applied to process the data, and the measurement data such as patients' age, serum Cys-C, RBP4, and NGAL levels were expressed as mean ± standard deviation ($\bar{x}\pm s$); analysis of variance (*F*-test) was used between the three groups, the *t*-test was used for comparison between two groups, the *Q*-test was used for normally distributed measures, and the rank sum test was used for nonnormally distributed measures. Categorical information was expressed as (*n*, (%)), using the chi-square test. Correlation between the two was performed using Pearson correlation analysis. Receiver Operating Characteristic (ROC) was plotted, and the area under the curve (AUC) was calculated to determine the diagnostic value of serum markers; AUC ≥0.700 suggested a high diagnostic value, the best cutoff value was calculated, and the specificity and sensitivity were determined. *P* < 0.05 was considered a statistically significant difference.

## 3. Results

### 3.1. Comparison of Baseline Information between the AKI Group and Healthy Group

The results of the comparison of baseline data between the two groups showed no statistically significant differences between the AKI group and the healthy group in terms of gender, age, and weight (*P* > 0.05). Serum Cys-C, RBP4, NGAL, and Scr levels were significantly higher in the AKI group than in the healthy group (*P* < 0.05) (Table 1).

### 3.2. Comparison of Serum Cys-C, RBP4, and NAGL Levels in Patients with Different Degrees of Traumatic AKI

After statistical analysis of serum Cys-C, RBP4, and NAGL levels in patients with different AKI conditions, we found that serum Cys-C, RBP4, and NAGL concentrations increased as the severity of the disease increased. The concentrations of all three serum markers in patients with different conditions showed AKI phase I < AKI phase II < AKI phase III, and the differences between the two were statistically significant (*P* < 0.05, Figure 1), which indicated that there was a relationship between all three serum markers and patients' conditions.

### 3.3. Correlation Analysis of Serum Cys-C, RBP4, and NAGL Levels and Serum Scr Concentration

We used the Pearson model to analyze the correlation between the two, and the results showed that serum Cys-C, RBP4, and NAGL levels were positively correlated with serum Scr concentration (their *r* values were 0.417, 0.341, and 0.474, respectively, *P* < 0.001, Figure 2), which indicated that all three serum markers could be used as indicators to evaluate patients' condition.

### 3.4. Diagnostic Value of Serum Cys-C, RBP4, and NAGL Alone and in Combination for the Diagnosis of Traumatic AKI

We used ROC curves to analyze the diagnostic value of serum markers for traumatic AKI disease and showed that the diagnostic values of serum Cys-C, RBP4, and NAGL alone and in combination were 0.769, 0.747, 0.771, and 0.905, respectively (Figure 3). To determine the optimal cutoff value for the diagnosis of fracture traumatic shock, the intersection point between the sensitivity and the 100-specificity curves of serum Cys-C, RBP4, NAGL, and “Cys-C + RBP4 + NGAL” was used. When the optimal cutoff values of serum Cys-C, RBP4, NAGL, and “Cys-C + RBP4 + NGAL” were 0.498, 0.451, 0.429, and 0.773, respectively, their sensitivities were 59.80%, 75.90%, 66.70%, and 86.20%, respectively, and their specificities were 91.10%, 73.30%, 88.90%, and 91.10%, respectively (Table 2). Among them, Cys-C + RBP4 + NGAL assay had the highest AUC, and the sensitivity and specificity were in the high range, which indicates that the combined assay of the three is of high clinical value for the diagnosis of traumatic AKI.

## 4. Discussion

Traumatic AKI can be caused by conditions such as crush syndrome, acute lung injury/acute respiratory distress syndrome (ALI/ARDS), and trauma-induced hypovolemic shock [12]. The degree and changes in renal injury can have an impact on the prognosis of patients with traumatic diseases, so early diagnosis of the patient's renal function status is particularly important. Measurement of serum urea nitrogen and Scr levels are currently important indicators for detecting deterioration in renal function, but the rise in Scr levels usually occurs 24 h after the onset of AKI and is easily influenced by gender, protein intake, and muscle metabolism, which does not allow for a timely diagnosis of AKI, making it necessary to find other more sensitive serum markers for the assessment of renal function [13].

Cys C is synthesized and secreted into the blood at a relatively constant rate in nucleated cells in the body, with a constant daily secretion, and is completely filtered by the glomerulus and taken up by the proximal tubule. The concentration of Cys C in the blood is determined only by the glomerular filtration rate and is not affected by physiological and pathological factors such as age and inflammation, so it can be used as a sensitive indicator to assess glomerular and tubular lesions [14, 15]. As an indicator that can also reflect the function of glomeruli and tubules, RBP4 is getting more and more attention in clinical practice, and it was mainly used as a screening marker for diabetic nephropathy and attracted attention in the early stage [16]. RBP4 is mainly synthesized by hepatocytes and is produced at a constant rate, and most of it can be reabsorbed by the renal tubules after passing through the glomerular filtration membrane, so the concentration of RBP4 in the blood is less affected by other factors when it is under normal physiological conditions [17]. Gonzalez-Calero et al. [18] showed that patients showed a significant increase in urinary RBP4 after the onset of AKI, and monitoring RBP4 has a positive role in the evaluation of the condition and prognosis of patients with AKI. NGAL plays an important role in immune defense, tumor development, and inflammatory immune response, and it also exerts a protective effect on the kidney through various mechanisms [19]. Under normal physiological conditions, NGAL has stable low expression in a variety of organs, including the bone marrow, stomach, and colon. A study by Lumlertgul et al. [20] found that, in patients with renal impairment, NGAL values were well outside the normal range values while serum creatinine was still in the normal range, which suggests that NGAL has a high application value for early diagnosis of AKI.

In this study, we found that serum Cys C, RBP4, and NGAL levels were higher in patients with traumatic AKI than in healthy patients and increased with the severity of the disease. To analyze the reasons for this, the impairment of glomerular filtration rate function and reduced tubular reabsorption after the onset of AKI leads to the retention of Cys C and RBP4 in the blood [21, 22]. When AKI occurs in patients with severe trauma due to insufficient effective circulation and other reasons, NGAL will be rapidly and efficiently expressed in renal tubular epithelial cells and is manifested by high NGAL levels in blood and urine [23]. Therefore, serum Cys C, RBP4, and NGAL levels were significantly altered in patients with traumatic AKI compared to the healthy population. After correlation analysis, we found that serum Cys C, RBP4 and NGAL levels were positively correlated with serum Scr levels, which suggests that Cys C, RBP4, and NGAL are potentially associated with the pathological process of kidney injury in patients with traumatic diseases, and their detection can help determine the renal function of patients. In order to explore the diagnostic value of the three in patients with traumatic AKI, the further ROC curve analysis was performed. The results showed that the serum Cys C, RBP4, and NGAL single detection and the three combined detection all have a certain diagnostic value (AUC > 0.700), and the AUC of the three combined detection is the highest. It can be seen that the detection of serum Cys C, RBP4, and NGAL alone has certain reference significance in the diagnosis of traumatic AKI, but the combined detection of the three has higher clinical value.

Overall, the severity of disease in patients with traumatic AKI was positively correlated with serum Cys C, RBP4, and NGAL levels, which suggests that these three serum markers can be used as indicators to evaluate the patient's condition. Compared with serum Cys C, RBP4, and NGAL alone, the combined test of the three has a higher application in the clinical diagnosis of traumatic AKI.

## Figures and Tables

**Figure 1:** Comparison of serum Cys-C, RBP4, and NAGL levels in patients with different degrees of traumatic AKI. (a) Comparison of serum Cys-C levels in AKI phase I, phase II, and phase III. (b) Comparison of serum RBP4 levels. (c) Comparison of serum NGAL levels. (d) Comparison of serum Scr levels. Compared with AKI phase I, ^*∗*^*P* < 0.05; compared with AKI phase II, ^∧^*P* < 0.05.

**Figure 2:** Correlation analysis of serum Cys-C, RBP4, NAGL levels, and serum Scr concentration. (a) Correlation analysis of serum Cys-C level and serum Scr concentration; the correlation between them both is positive, *r* = 0.417, *P* < 0.001. (b) There is a positive correlation between serum RBP4 and serum Scr concentration, *r* = 0.341, *P* < 0.001. (c) There is a positive correlation between serum NGAL and serum Scr concentration, *r* = 0.474, *P* < 0.001.

**Figure 3:** ROC curve of the diagnostic value of serum Cys-C, RBP4, and NAGL alone and combined detection of traumatic AKI. (a) ROC curve of serum Cys-C, AUC = 0.769. (b) ROC curve of serum RBP4, AUC = 0.747. (c) ROC curve of serum NGAL, AUC = 0.771. (d) ROC curve of combined detection of serum Cys-C, RBP4, and NGAL, AUC = 0.905.

**Table 1:** Comparison of general data of the AKI group and Health group.

Data	AKI group (*n* = 132)	Health group (*n* = 130)	*P* value
Gender (*n*, %)			0.770
Male	83 (62.88)	84 (64.62)	
Female	49 (37.12)	46 (35.38)	
Age, mean (SD), year	43.24 ± 9.23	42.06 ± 7.13	0.248
Weight, mean (SD), kg	63.23 ± 6.87	64.09 ± 7.02	0.317
Cys-C, mean (SD), mg/L	3.49 ± 1.81	0.75 ± 0.28	<0.001
RBP4, mean (SD), mg/L	60.47 ± 25.93	25.58 ± 3.12	<0.001
NGAL, mean (SD), ng/mL	152.10 ± 89.66	24.46 ± 8.23	<0.001
Scr, mean (SD), *μ*mol/L	235.61 ± 72.29	57.26 ± 20.13	<0.001

**Table 2:** Analysis of the diagnostic value of serum Cys-C, RBP4, and NAGL alone and in combination for traumatic AKI.

Index	AUC	95% confidence interval	Cutoff	Sensitivity (%)	Specificity (%)
Cys-C	0.769	0.690∼0.847	0.498	59.80	91.10
RBP4	0.747	0.664∼0.830	0.451	75.90	73.30
NGAL	0.771	0.693∼0.849	0.429	66.70	88.90
Cys-C + RBP4 + NGAL	0.905	0.852∼0.958	0.773	86.20	91.10

## Data Availability

The data used during the current study are available from the corresponding author on reasonable request.
